# Effect of the COVID-19 pandemic on the mental health, daily and occupational activities of pediatric otolaryngologists in Latin America

**DOI:** 10.3389/fpubh.2022.735073

**Published:** 2022-10-20

**Authors:** Augusto Peñaranda, Sergio Moreno-López, Daniel Peñaranda, Lucía C. Pérez-Herrera

**Affiliations:** ^1^Otolaryngology and Allergy Research Groups, Unidad Médico Quirúrgica de Otorrinolaringología (UNIMEQ-ORL), Bogotá, Colombia; ^2^School of Medicine, Universidad de Los Andes, Bogotá, Colombia; ^3^Department of Otolaringology, Fundación Santa Fe de Bogotá, Bogotá, Colombia; ^4^Department of Otolaryngology, Fundación Universitaria de Ciencias de la Salud-Hospital de San José, Bogotá, Colombia

**Keywords:** anxiety, depression, stress, COVID-19, otolaryngologists

## Abstract

**Background:**

Otolaryngologists have a higher risk of physical/psychological problems due to their frequent exposure to SARS-CoV-2. There is no information about the impact of COVID-19 on the mental health of these specialists in low/middle-income countries from Latin America. This study aimed to assess the frequency of anxiety, depression, and stress, as well as the changes in occupational and daily activities due to the COVID-19 pandemic in a group of pediatric otolaryngologists in Latin America.

**Methods:**

Observational, cross-sectional study conducted between October and December 2020. Mental health tools such as the Generalized Anxiety Disorder−7, the Patient Health Questionnaire-9, and the Perceived Stress Scale-10 were applied. Fear to COVID-19 scale and questionnaires about occupational and daily activities were also applied.

**Results:**

Among 55 pediatric otolaryngologists, the frequency of anxiety, depression, and stress were 67.3%, 45.5, and 40%, respectively. Up to 27.3% of the specialists reported moderate to severe symptoms of anxiety, while 7.3 and 40% presented moderate depression and stress symptoms. The specialists reported a reduction of 58.3% of their consultations, as well as a 51.7% reduction in their monthly income compared to the same period before the pandemic. Up to 14.6% of the specialists expect to incorporate long-term (>1 year) drastic changes in their daily activities due to the pandemic.

**Conclusions:**

The frequency of anxiety, depression, and stress was high among pediatric otolaryngologists in Latin America compared to previous studies performed in high-income countries. Further research on these psychological outcomes is needed to achieve early mental health strategies.

## Introduction

The Severe Acute Respiratory Syndrome Coronavirus-2 (SARS-CoV-2) pandemic has significantly disrupted Latin American health care systems (1). High mortality rates due to coronavirus disease-2019 (COVID-19) have been reported, and there are significant challenges in access to vaccination in most low/middle-income countries (2). Otolaryngologists who perform aerosol-generating procedures are frequently exposed to high viral loads of SARS-CoV-2 in the respiratory mucosa (3, 4). Thus, these specialists have a higher risk of developing physical and psychological problems due to the COVID-19 pandemic. A current study assessing the psychological outcomes in otolaryngologists in the United States during the COVID-19 pandemic showed that anxiety, distress, and depression were reported in 47.9, 60.2, and 10.6% of this population, respectively (5). This study highlighted that institutions should start focusing on the mental well-ness of these specialists, and further studies are needed to capture a longitudinal picture of this scenario (5).

Furthermore, routine medical practice has been severely disrupted by the pandemic, leading to several changes in the way otolaryngologists provide care (6–8). Practices such as telehealth underwent a significant expansion, and although it may not be viable for all patients, it has proven beneficial in specific circumstances (7). The adjustment issues related to these changes in the clinical practice could also trigger adverse psychological outcomes in these specialists (9). To date, no has study described the changes in occupational and daily activities due to the COVID-19 pandemic in pediatric otolaryngologists, and there is no information about the mental health of these specialists in Latin America. There are only two studies in the English literature assessing the psychological outcomes in otolaryngologists from Latin America (10, 11). This information is essential to achieve early mental health strategies and to prevent long-lasting implications. The impact of the pandemic on the psychological well-being of medical staff in low/middle-income countries is yet to be established. This study aimed to describe the frequency of depression, anxiety, and stress, as well as the changes in occupational and daily activities among pediatric otolaryngologists during the COVID-19 pandemic in Latin America.

## Methods

### Study design

This was an observational, cross-sectional study aimed to determine the frequency and associated factors of anxiety, depression, and stress in pediatric otolaryngologists during the COVID-19 pandemic in Latin America. The study was conducted using self-administered, anonymous online surveys to collect sociodemographic and mental health questionnaires from October to November 2020. Internationally validated questionnaires such as the Generalized Anxiety Disorder−7 (GAD7), the Patient Health Questionnaire-9 (PHQ9), and the Perceived Stress Scale-10 (PSS10) were used to determine the frequency of anxiety, depression, and stress. A sociodemographic questionnaire including a Fear to COVID-19 scale was also applied. The specialists were invited to participate either through social networks and/or through an e-mail invitation sent to a society of pediatric otolaryngologists from Latin America. If the participants accepted, they proceeded to complete the questionnaires in the KoBoToolbox platform. Ethics committee approval was received from the ethics committee of the Hospital Universitario Fundación Santa Fe de Bogotá (CCEI-12489-2020) according to the Helsinki Declaration. Informed Consent was obtained from all the participants. No incentives were offered for study participation, and participants were allowed to finish the survey at any time.

### Study population

The study population included specialists who belonged to a group of pediatric otolaryngologists from Latin America and conducted in-person consultations and/or telemedicine. Exclusion criteria were specialists who reported a prior diagnosis of mental health disorders confirmed by a psychiatrist or mental health professional, and those who reported any acute/chronic condition that could limit their ability to answer the questionnaires. Regarding the sample selection method, a non-probabilistic snowball sampling was conducted, and a power calculation was performed based on a prior study by Perez-Herrera et al. (11) considering that this assessment showed a medium to high confidence level in terms of type II error. A pilot test was performed including 5 Colombian otolaryngologists, and two additional questions were included in the sociodemographic questionnaire.

### Mental health questionnaires

Symptoms of anxiety, depression, and stress were assessed by applying the validated Spanish versions of the GAD-7, PHQ-9, and PSS-10, respectively (12–14). The GAD-7 questionnaire assesses symptoms of anxiety over the past 2 weeks classified as normal (0–4), mild (5–9), moderate (10–14), and severe (15–21) anxiety. As priorly stated by the Spanish validation of GAD-7, the cutoff point used for General Anxiety Disorder was 10 points (12). Moreover, to establish this cut-off point as criteria to assess the symptoms of anxiety, a Spanish validation of the GAD-7 in a Latin American population that reported good reliability (Cronbach = 0.920) was also considered (15). The PHQ-9 assesses depression symptoms classified as none (0–4), mild (5–9), moderate (10–14), moderately severe (15–19), severe (20–27). The cutoff point for major depression was a total score of ≥10 as priorly established by a Spanish validation of this questionnaire in a Latin American population (Cronbach α = 0.89) (13). Finally, the PSS-10 questionnaire assesses the perception of stressful experiences during the preceding month and the total score can be classified as low-stress (0–13), moderate-stress (14–26), and high-perceived stress (27–40) (14, 16). The Spanish version of the PSS-10 questionnaire has been priorly validated and adapted in Latin American populations and showed good reliability (Cronbach α = 0.78) (17).

### Variables related to COVID-19, and changes in occupational and daily activities questionnaires

A “Fear score of COVID-19” ordinal questionnaire ranging from 1 to 5 (1: No fear at all, 5: utmost fear) was applied to assess the fear of contagion, fear of the possibility of a negative outcome (death/sequelae), as well as the fear of infecting a family member and/or friends. The questionnaire about the occupational activities of these specialists was developed by the authors of this manuscript and assessed the following items: number of years of work experience, number of hours worked per week, work mode (In-person consultation/Telemedicine), changes in the income and reduction in consultation during the last 6–8 months compared to the same period before the pandemic, whether the protection elements were by their employer, and the most frequent protection elements used in their consultations during the pandemic. Furthermore, a questionnaire on when the specialists would expect to resume their daily activities considering the scenario of the COVID-19/ SARS-CoV-2 pandemic was applied. This questionnaire was developed by “The New York Times” and previously applied to 511 epidemiologists (18). These answers only reflect their individual life circumstances and opinions and should not be used as guidelines for the public.

### Statistical analysis

Statistical analysis was performed using Stata 16MP software (StataCorp, College Station, TX, USA). All the frequencies and percentages were calculated for the qualitative variables and central tendency and dispersion measures were estimated for the quantitative variables. The frequency of symptoms of anxiety, depression, and stress was also calculated. Finally, a Hierarchical clustering on principal components was performed to describe probable joint relationships of anxiety, stress, and depression considering the country of the participants, and the variables related to COVID-19 included in the study. An exploratory analysis of factors associated with anxiety, depression, and stress was also performed based on a Poisson regression model with robust errors to estimate the prevalence ratio (PR) of the sociodemographic and clinical variables related with COVID-19. We hypothesized that a higher prevalence of psychological outcomes would be found in the population that reported higher scores on the fear to COVID-19 scale. All the variables with biological plausibility were included in the model, and the goodness of fit was assessed with a linear test. The level of significance was priorly established as 5%.

## Results

A total of 55 individuals were included, of which 52.7% (*n* = 29) of them were older than 50 years old. The median length for solving the questionnaires was 24 min (IQR = 19–36). The baseline demographic characteristics of the study population are described in Table 1. Up to 92.5% (*n* = 51) of the study population performed in-person consultation. Overall, 34.6% (*n* = 19) of the specialists considered that the personal protection elements provided by their employer were not enough to prevent COVID-19 infection. Among the most frequent biosafety elements used in their clinical practice were surgical masks with 52.7% (*n* = 29), and N95 respirators with 38.2% (*n* = 21). Most of the specialists were from Mexico (27.3%, *n* = 15), Argentina (25.5%, *n* = 14), and Venezuela (20%, *n* = 11).

**Table 1:** Baseline demographic and occupational characteristics of the study population.

**Variables**	**Participants *n* = 55**	
	***n***	**%**
Sex. Female/Male	30/25	54.6/45.4
Age in years ^(a)^	49.8 (10.6)	50.5 (39.8–57.6)
Age group		261
30 to 40 years-old	14	25.5
40 to 50 years-old	12	21.8
50 to 60 years-old	18	32.7
More than 60 years-old	11	20.0
Marital status		
Married/Free union	43	78.2
Divorced/widowed	2	3.6
Single or other	10	18.2
Country		
Mexico	15	27.3
Argentina	14	25.5
Venezuela	11	20.0
Chile	4	7.3
Costa Rica	4	7.3
Colombia	2	3.6
Perú	2	3.6
Honduras	1	1.8
Nicaragua	1	1.8
Paraguay	1	1.8
Years of work experience ^(a)^	20.5 (11.1)	22 (10–29)
Number of hours worked per week ^(b)^	30 (18–50)
Work mode		
In-person consultation	51	92.7
Telemedicine	27	49.1
The income during these 6–8 months compared to the same period before the pandemic		
Has increased	7	12.7
Has decreased	41	74.6
Remains the same	7	12.7
Percentage reduction in consultation during the pandemic ^(a)^	58.3 (19.3)	60 (50–70)
Percentage reduction of your monthly income ^(a)^	51.7 (22.2)	50 (40–70)
¿Are the protection elements provided by your employer enough?		
No	19	34.6
¿Did you have to buy your personal protection elements from your “own pocket” expenses?		
Yes	31	56.4
¿Which of the following personal protection elements do you use in your clinical practice?		
Surgical mask	29	52.7
N95 respirator	21	38.2
Surgical gloves	19	34.6
Face masks	13	23.6
Face shields or glasses	11	20.0

Values are expressed in Mean (SD) and Median (p25–p75).

Values are expressed in Median (p25–p75).

### Frequency and severity of psychological disorders

Table 2 shows the frequency and severity of depression, anxiety, and stress in the study population. Overall, the frequency of anxiety was higher than the frequency of depression or stress in the study population. The frequency of anxiety, depression, and stress were 67.3, 45.5, and 40%, respectively. Up to 27.3% of the specialists reported moderate to severe symptoms of anxiety, while 7.3 and 40% presented moderate symptoms of depression and stress, respectively.

**Table 2:** Frequency and severity of depression, anxiety, and stress in the population.

**Condition**	**Participants (*n* = 55)**	
	***n***	**%**
**Anxiety**	37	67.3
**Depression**	25	45.5
**Stress**	22	40.0
**Anxiety in comorbidity with**		
•Depression	24	43.6
•Stress	21	38.2
**Depression in comorbidity with Stress**	16	29.1
**GAD7: Anxiety severity scores**		55
Normal	18	32.7
Mild	22	40.0
Moderate	11	20.0
Severe	4	7.3
**PHQ9: Major depression severity scores**		261
None	30	54.6
Mild	21	38.2
Moderate	4	7.3
**PSS10: Stress severity scores**		261
Low	33	60.0
Moderate	22	40.0

### Variables related to COVID-19

By the time of this study (October-November 2020), 3.6% (*n* = 2) of the participants had been diagnosed with a positive infection of SARS-CoV-2 and 23.6% (*n* = 13) had been isolated on suspicion of infection with COVID-19. Around 83.6% (*n* = 46) reported being afraid of contagion by COVID-19, and 96.4% (*n* = 53) were afraid of the possibility of infecting their family and/or friends. The “Fear scores” of COVID-19 were higher regarding the possibility of infecting a family member and/or friends compared with their infection. These results are listed in Table 3.

**Table 3:** Variables related to COVID-19.

**Variable**	**Participants (*n* = 55)**	
	***n***	**%**
**Variables related to COVID-19**		
**Factors associated with contagion**		
Frontline health worker	52	94.6
Close contact with a positive case of COVID-19	8	14.6
None	2	3.6
**Have you been diagnosed with COVID-19 infection?**
Yes	2	3.6
**Have you been isolated on suspicion of infection with COVID-19 infection?**
Yes	13	23.6
**Any of the following family members had been diagnosed with COVID-19?**		
Father/Mother	1	1.8
Brother/sister	5	9.1
Son	6	10.9
Partner/Couple	2	3.6
**Have you been afraid of COVID-19 contagion?**		
Yes	46	83.6
**Have you been afraid of the possibility of a negative outcome (death/sequelae) due to COVID-19?**		
Yes	46	83.6
**Have you been afraid of infecting your family and/or friends with COVID-19?**		
Yes	53	96.4
**COVID-19 Fear score (On a scale from 1 to 5):**		
Fear of contagion ^(a)^	3.5 (3-4)
Negative outcome (death. sequelae) ^(a)^	4 (3–4)
Infect a family member and/or friends ^(a)^	4.5 (3–5)

Values are expressed in Mean (SD) and Median (p25–p75).

### Changes in occupational and daily activities due to COVID-19

The changes in occupational activities are described in Table 1. The specialists reported a reduction of 58.3% of their consultations, as well as a 51.7% reduction in their monthly income compared to the previous 6–8 months before the pandemic. Up to 34.5% of the specialists reported that their employer did not provide the protection elements needed for their consults, and 56.4% reported that they had to buy these elements from their own expenses. Moreover, Table 4 describes the daily activities that the specialists expect to resume considering the scenario of the Covid-19/ SARS-CoV-2 pandemic. Specialists reported they would never meet again with someone they don't know well (20%), bring in the mail without precautions (18.2%), stop routinely wearing a face mask (14.5%), attend a church or other religious service (12.7%), exercise at a gym or fitness studio (12.7%), work in a shared office (10.9%), or ride a subway/bus (10%). Up to 14.55% of the specialists expect to incorporate long-term (>1 year) drastic changes in their daily activities due to the pandemic.

**Table 4:** Daily activities the specialists expect to resume considering the scenario of the Covid-19/ SARS-CoV-2 pandemic.

**Variables**	**Total** ***n* =** **5**		**Variables**	**Total** ***n* =** **55**		**Variables**	**Total** ***n* =** **55**	
	***n***	**%**		***n***	**%**		***n***	**%**
Attend a sporting event. concert or play		261	Get a haircut at a salon or barbershop			Hug or shake hands when greeting a friend		
<3 months	2	3.6	<3 months	25	45.5	<3 months	10	18.2
3 to 12 months	22	40.0	3 to 12 months	18	32.7	3 to 12 months	24	43.6
> 1 year	28	50.9	> 1 year	5	9.1	> 1 year	14	25.5
Never again	2	3.6	Never again	5	9.1	Never again	4	7.3
Does not apply	1	1.8	Does not apply	2	3.6	Does not apply	3	5.5
Attend a wedding or a funeral			Eat at a dine-in restaurant			Go out with someone you don't know well		
<3 months	4	7.2	<3 months	16	29.1	<3 months	3	5.5
3 to 12 months	16	29.1	3 to 12 months	30	54.6	3 to 12 months	14	25.5
> 1 year	30	54.6	> 1 year	7	12.7	> 1 year	17	30.9
Never again	3	5.5	Never again	1	1.8	Never again	11	20.0
Does not apply	2	3.6	Does not apply	1	45.5	Does not apply	10	18.2
Attend a small social event or dinner with a small group of people			Attend a church or other religious service			Stop routinely wearing a face mask		
<3 months	22	40.0	<3 months	10	18.1	<3 months	1	1.8
3 to 12 months	25	45.5	3 to 12 months	25	45.5	3 to 12 months	11	20.0
> 1 year	4	7.3	> 1 year	8	14.6	> 1 year	33	60.0
Never again	3	5.5	Never again	7	12.7	Never again	8	14.6
Does not apply	1	1.8	Does not apply	5	9.1	Does not apply	2	3.6
See a doctor for a non-urgent appointment			Send kids to school. camp or day care			Bring in mail without precautions		
<3 months	27	49.1	<3 months	5	9.1	<3 months	10	18.2
3 to 12 months	11	20.0	3 to 12 months	24	43.6	3 to 12 months	17	30.9
> 1 year	2	3.6	> 1 year	12	21.8	> 1 year	17	30.9
Never again	4	7.3	Never again	2	3.6	Never again	10	18.2
Does not apply	3	5.5	Does not apply	11	20.0	Does not apply	1	1.8
Exercise at a gym or fitness studio			Work in a shared office			Travel by airplane		
<3 months	12	21.8	<3 months	13	23.6	<3 months	9	16.4
3 to 12 months	20	36.4	3 to 12 months	25	45.5	3 to 12 months	28	50.9
> 1 year	13	23.6	> 1 year	3	5.5	> 1 year	14	25.5
Never again	7	12.7	Never again	6	10.9	Never again	3	5.5
Does not apply	3	5.5	Does not apply	8	14.6	Does not apply	1	1.8
Ride a subway or a bus			Send children on play dates			Go on vacations overnight		
<3 months	9	16.4	<3 months	17	30.9	<3 months	8	14.6
3 to 12 months	15	27.3	3 to 12 months	14	25.5	3 to 12 months	30	54.6
> 1 year	16	29.1	> 1 year	9	16.4	> 1 year	13	23.6
Never again	10	18.2	Never again	2	3.6	Never again	4	7.3
Does not apply	5	9.1	Does not apply	13	23.6	Does not apply	0	0.00
Hike or picnic outdoors with friends			Visit elderly relative or friend in their home			Do you expect to incorporate long-term (>1 year) drastic changes in your daily activities due to the pandemic?		
<3 months	24	43.6	<3 months	18	32.7	Yes	8	14.6
3 to 12 months	20	36.4	3 to 12 months	23	41.8			
> 1 year	4	7.3	> 1 year	10	18.2			
Never again	5	9.1	Never again	1	1.8			

### MCA: Joint characteristics of anxiety, depression, and stress

Figure 1 shows the MCA among the mental health outcomes, the country of the participants, and the variables related to COVID-19 included. The clusters (triangles) shaped in the spatial distribution show the associations between categorical variables, and the variables that are closer to each other in the MCA show significant statistical associations between them. Cluster # 1 showed that anxiety, stress, and depression were most frequently found in: women (*p* < 0.05), participants that reported their fear of the possibility of a negative outcome due to COVID-19 (*p* < 0.05), and those participants who performed in-person consultations (*p* < 0.05). Cluster # 2 grouped participants who were practicing teleworking (*p* < 0.01) and were not afraid of infecting a friend/family member (*p* < 0.01). Finally, cluster #3 showed that the participants who did not report anxiety, stress, or depression were mostly from Costa Rica (*p* < 0.05), and these participants were not afraid of a possible death/sequel due to COVID-19 (*p* < 0.01).

**Figure 1:** Cluster analysis of the variables associated with the mental health outcomes. The variables showed a distribution in three groups (designated in an *ad hoc* way in this figure).

### Factors associated with symptoms of anxiety, depression, and stress

Factors associated with anxiety, depression, and stress are shown in Table 5. Anxiety (PR: 1.33; 95%CI: 1.07–1.65) and depression (PR: 1.94; 95%CI: 1.29–2.92) were more frequently found in specialists who reported fear of contagion of COVID-19. A higher frequency of stress was found in female specialists (PR: 2.39; 95%CI: 1.12–5.07).

**Table 5:** Factors associated with symptoms of anxiety, depression, and stress.

**Variable ^h^**	**Anxiety (GAD 7)**				**Depression (PHQ 9)**				**Stress (PSS 10)**			
	**Multivariate model ^a^**		**Reduced model ^b^^,^^g^**		**Multivariate model ^c^**		**Reduced model ^d^^,^^g^**		**Multivariate model ^e^**		**Reduced model ^f^^,^^g^**	
	**PR**	**95%CI**	**PR**	**95%CI**	**PR**	**95%CI**	**PR**	**95%CI**	**PR**	**95%CI**	**PR**	**95%CI**
Age in years	0.98	0.96– 1.00	—	—	0.99	0.95–1.03	—	— —	0.98	0.94–1.03	—	—
Female sex	1.37	0.88–2.13	1.34	0.89-2.02	1.39	0.70–2.75	1.06	0.59–1.90	2.42	1.07–5.49	**2.39**	**1.12−5.07**
Marital status			—	—			—	—			—	—
Divorced/widowed/single/other	0.82	0.48–1.41			0.73	0.24– 2.23			1.06	0.42– 2.69		
Telemedicine			—	—			—	—			—	—
Yes	0.80	0.50–1.28			0.68	0.33–1.40			0.92	0.43–1.95		
The protection elements provided by your employer are enough?			—	—			—	—			—	—
Yes	1.13	0.69–1.86			0.71	0.35–1.44			0.71	0.33–1.54		
Have you been diagnosed with COVID-19 infection?											—	—
Yes	1.77	0.99–3.17	**1.33**	**1.07-1.65**	1.80	0.77–4.20	**1.94**	**1.29–2.92**	0.34	0.04–2.98		
Have you been afraid of COVID-19 contagion?			—	—			—	—			—	—
Yes	1.28	0.65–2.55			0.80	0.36–1.78			0.77	0.34–1.74		
Have you been afraid of the possibility of a negative outcome (death/sequelae) due to COVID-19?			—	—								
Yes	1.43	0.64–3.17			5.00	0.72–34.87	4.54	0.70–29.52	5.52	0.84– 36.05	4.59	0.73–28.80
Number of hours worked per week	1.00	1.00–1.00	—	—	1.00	1.00–1.00	—	—	1.00	1.00–1.00	—	—
Percentage reduction in consultation during the pandemic	0.99	0.99–1.00	—	—	0.99	0.98– 1.01	—	—	1.00	0.99– 1.02	—	—

a . Log-likelihood Intercept only, 46.712; Log-likelihood Model, 44.877; AIC, 111.754; BIC, 132.787;

b . Log-likelihood Intercept only, 51.667; Log-likelihood Model, 51.159; AIC, 106,318; BIC, 110.332;

c . Log-likelihood Intercept only, 40.062; Log-likelihood Model, 37.165; AIC, 96.331; BIC, 117.363;

d . Log-likelihood Intercept only, 44.711; Log-likelihood Model, 42.437; AIC, 90.847; BIC, 96.895;

e . Log-likelihood Intercept only, 38.326; Log-likelihood Model, 34.538; AIC, 91.076; BIC, 112.109;

f . Log-likelihood Intercept only, 42.158; Log-likelihood Model, 38.831; AIC, 83.662; BIC, 89.684;

g . The reduced model was based on the Furnival-Wilson leaps-and-bounds algorithm/stepwise methodology, link test p>0.05; h. Bolded numbers highlight the significant associations between the variables.

## Discussion

The Latin American pediatric otolaryngologists included in this study reported high levels of anxiety (67.3%), depression (45.5%), and stress (40%) symptoms. The frequency of these psychological outcomes was even higher than that reported by a prior study in otolaryngologists from high-income countries during the pandemic (anxiety: 47.9%, depression: 10.6%, and distress: 60.2%) (5). During the pandemic, the highest levels of anxiety, depression, and stress in Latin American otolaryngologists were recently reported in Colombia (56.1, 28.1, and 28.1%, respectively) (11). Prior to the pandemic, the weighted mean frequency of anxiety and affective disorders in the general population from Latin America vs the general population in North America was: 13.2 vs. 16.7%, and 7.7 vs. 9.1%, respectively (19). Nevertheless, there is no data about these psychological outcomes in Latin American healthcare workers before the pandemic, and healthcare workers are more susceptible to develop adverse psychological outcomes due to overburdened workload, inefficiencies in medical records, and broken health care systems (20, 21). Moreover, several authors describe a significant raise in the levels of depression and anxiety worldwide due to isolation, lockdown, and physical distancing related to the pandemic (22, 23). This should be considered for the interpretation of the results.

This study was performed in medical specialists who are exposed to high viral loads of the nasal mucosa and respiratory tract (8, 24, 25), this setting could also account for the higher frequency and severity of psychological outcomes. Up to 27.3% of the specialists reported moderate to severe symptoms of anxiety, while 7.3 and 40% presented moderate symptoms of depression and stress. Likewise, anxiety (PR: 1.33; 95%CI: 1.07–1.65) and depression (PR: 1.94; 95%CI: 1.29–2.92) were more frequently found in specialists who reported fear of contagion of COVID-19, which highlights that these symptoms could be related to an adjustment response to the pandemic. Focusing on healthcare worker's mental health is essential considering that the rates of adverse psychological outcomes raised due to the COVID-19 pandemic. Civantos *et al* stated that depending on the trajectory of the pandemic, the mental health symptoms of healthcare workers could intensify or diminish over time (5). Thus, during the last months of 2020, the psychological outcomes could have increased along with the shortage of personal protective equipment, and the physical and emotional exhaustion related to the epidemic peak outbreak. Studies addressing these psychological outcomes in different time points of the COVID-19 pandemic on low/middle-income populations are needed.

A higher frequency of stress was found in female specialists (PR: 2.39; 95%CI: 1.12–5.07), which has been similarly reported by prior studies during the pandemic (26, 27). The pediatric otolaryngologists included in this study reported a reduction of 58.3% (SD: 19.2) on their consultations and a reduction of 51.7% (SD: 22.1) of their monthly income. Anxiety could be related to the fear of COVID-19 and could be increased by an income reduction considering the decrease in consultations and otolaryngology elective surgical procedures. A prior study in the United States described that a significant decrease in household income is associated with an increased risk of incident mood, or anxiety disorders (adjusted OR: 1.3; 99% CI: 1.1–1.6) (28). This could account for the high levels of anxiety and depression disorders found in this population. On the other hand, a systematic review and meta-analysis by Pappa *et al* stated that these physical and mental adverse outcomes could be triggered by inadequate personal equipment, nosocomial transmission, and the need to make ethically difficult decisions (21). Up to 34.6% of the otolaryngologists reported their concern regarding inadequate personal protective equipment which is noteworthy considering their risk standing on the front-line of the pandemic. This issue could trigger physical and mental adverse outcomes and could increase the fears related to SARS-CoV2 contagion (21). Moreover, the fear score of the possibility of infecting family and/or friends (media*n* = 3.5; IQR: 3–4) was higher than the fear of their own infection (media*n* = 4.5; IQR: 3–4). Despite the high levels of anxiety related to those fears, these findings highlight the awareness and social responsibility of the medical staff. Overall, our findings stand out the imperative need to provide early mental health interventions and support in healthcare workers, particularly high-risk specialists such as otolaryngologists to prevent long-lasting implications.

COVID-19 pandemic transformed the daily activities of physicians. In our population, 23.6% had to undergo isolation because of either being infected by COVID-19 or being suspicious of infection. Prior authors state that healthcare workers' resilience could be compromised by isolation, as well as the loss of social support, and unsettling changes in the working setting (21). Drastic changes in daily leisure activities reported in this study could also worsen this scenario. About 16 to 24% of the population stated that they will “never again” resume daily activities. In addition to the occupational and income-related risk factors for adverse psychological outcomes, the radical changes in the daily and leisure activities of the healthcare workers could speed up the development of mental disorders. About the results showed by the MCA, we highlight that anxiety, stress, and depression were most frequently found in women and participants that reported their fear of the possibility of a negative outcome due to COVID-19. These results are similar to a prior Latin American mental health report that described a higher frequency of these outcomes in women (29). Besides, a prior study performed in Colombia that showed higher levels of mental health outcomes in otolaryngologists who expressed their fear of COVID-19 contagion (11). However, this is the first study that describes that anxiety, depression, and stress were more frequent in those participants who performed in-person consultations, and less frequent in those who practiced teleworking. This scenario highlights the importance of new technologies to improve the clinical practice of otolaryngologists.

Overall, most Latin American countries have historically invested less in mental health care compared to other subregions and countries of similar income (29). Preventive strategies to ensure minimal mental health conditions include adequate occupational environments, financial support, and ensuring adequate personal protection equipment and vaccination access. Psychological interventions to enhance psychological resilience and coping strategies, as well as institutional support, could be essential for reducing mental health disorders in healthcare professionals (30). Current analyses forecast a shadowy overview for health workers and people at risk from low to middle-income countries due to the access barriers for COVID-19 vaccination (2). Therefore, the investment in psychological and/or psychiatric support without occupational stigmatization should be granted to prevent long-term psychological consequences triggered by the pandemic.

Among the limitations of the study, we highlight that the data were obtained from a group of pediatric otolaryngologists from Latin America. This specialty was recently formed in Latin America, and there is no official information about the number of pediatric otolaryngologists (31). Despite we invited all the otolaryngologists registered in the Latin American Association of Pediatric Otolaryngology, the sample size could be more representative of Latin American population to obtain more robust results. We also stand out that non-probabilistic sampling is not the ideal path to obtain representativeness. Despite we performed a Poisson regression model to assess the associations between the variables, considering the small size of the sample these associations should be thoughtfully analyzed under an exploratory perspective. Due to the small sample size of the subgroups of specialists with depression and stress, we were not able to estimate the statistical models of associated factors with these outcomes. Moreover, we stand out that despite the Spanish versions of the psychological questionnaires were priorly validated in Latin American countries, some cultural values and differences among each specific country could lead to differences in the interpretation of the questionnaires, and this should be considered as an important limitation of the study. Further studies assessing associated factors, quality of life, and mental health in healthcare professionals especially in low to middle-income countries are needed. This information would be essential to support the development of preventive and therapeutic public health strategies needed to reduce anxiety, depression, and stress in health professionals, particularly in Latin America.

## Conclusions

High levels of anxiety, depression, and stress symptoms were found in this group of pediatric otolaryngologists. These levels were higher than those reported by a prior study in otolaryngologists from the United States during the COVID-19 pandemic. The specialists reported a significant reduction in their consultations and their monthly income. Preventive strategies to ensure minimal mental health conditions include adequate occupational environments, financial support, and ensuring adequate personal protection equipment and vaccination access. Psychological and/or psychiatric support without occupational stigmatization should be granted by the institutions.

## Data availability statement

The original contributions presented in the study are included in the article/supplementary material, further inquiries can be directed to the corresponding author.

## Ethics statement

The studies involving human participants were reviewed and approved by the Ethical Committee of the Hospital Universitario Fundación Santa Fe (Protocol Number: CCEI-12489-2020) approved this study. The patients/participants provided their written informed consent to participate in this study.

## Author contributions

Conceptualization, supervision, and funding acquisition: AP. Methodology: SM-L and AP. Software: SM-L. Formal analysis, investigation, writing—original draft and writing—review & editing: All authors contributed to this process. Data curation: LP-H and SM-L. All authors contributed to the article and approved the submitted version.

## Funding

This study was supported by the Unidad Medicoquirúgica de Otorrinolaringología (Unimeq-Orl), Bogotá, Colombia.

## Conflict of interest

The authors declare that the research was conducted in the absence of any commercial or financial relationships that could be construed as a potential conflict of interest.

## Publisher's note

All claims expressed in this article are solely those of the authors and do not necessarily represent those of their affiliated organizations, or those of the publisher, the editors and the reviewers. Any product that may be evaluated in this article, or claim that may be made by its manufacturer, is not guaranteed or endorsed by the publisher.
